This article has been retracted.

# Construction of a Legal System of Corporate Social Responsibility Based on Big Data Analysis Technology

**DOI:** 10.1155/2022/8448095

**Published:** 2022-10-07

**Authors:** Jiuzheng Pei

**Affiliations:** North China University of Water Resources and Electric Power, Zhengzhou 450000, China

## Abstract

The company is an essential organization in modern society, and the company has transformed from a purely economic organization to a corporate citizen that realizes economic responsibility and practices social responsibility at the same time. It is only by constructing a legal system of corporate social responsibility that companies can take social responsibility on the track of the legal system, realize the company's mission of the times, and achieve a win-win situation for both the company and society. This paper used the LDA and text clustering methods to analyze existing legal texts. It obtained the theme and text clustering results, thus proposing five aspects of the legal system construction framework to guide the corporate social responsibility legal system, which has pioneering significance.

## 1. Introduction

A distinctive feature of modern society is its great uncertainty and riskiness. The exposed crises in food safety, drug safety, environmental protection, network security, etc. have seriously affected the establishment of a harmonious society [1]. That is company creates these risks [2]. Companies have a unshirkable responsibility in these issues, and how to make companies achieve economic benefits while actively fulfilling their social responsibilities is a pressing issue in modern society. The company is an essential organization in modern society. In the past, it was defined as a purely economic organization, with the sole responsibility of creating profits to pay taxes and profits [3]. The immediate reason for the rise of corporate social responsibility thinking, theory, and practice is that “many companies disregard the rule of law and ethics in the pursuit of short-term profit maximization, or deliberately take advantage of the legal loopholes.” [4] With the development of society, companies have transformed from purely economic organizations to corporate citizens who realize economic responsibility and practice social responsibility at the same time. Improving the legal system and regulating the social responsibility of the company can make the company take more social responsibility. Corporate social responsibility (CSR) means that while creating profits and taking legal responsibilities to shareholders and employees, enterprises should also take responsibilities to consumers, communities, and the environment. Corporate social responsibility requires enterprises to go beyond the traditional idea of taking profits as the only goal. It emphasizes the importance of paying attention to the value of people in the production process, emphasizing the contribution to the environment, consumers, and society. The construction of the legal system of corporate social responsibility will enable the company to assume social responsibility on the track of the legal system, realize the company's mission of the times, and achieve a win-win situation for both the company and society [5].

In the past, the research on the construction of the legal system of corporate social responsibility was mainly based on theoretical and comparative studies, which explored the relatively mature concepts and theoretical foundations of corporate social responsibility at home and abroad [6]. It analyzed the basic principles and legislative contents of the legislation on the corporate social responsibility legal system. Manual analysis is not objective, scientific, and comprehensive [7]. When conducting manual analysis, there are problems such as significant differences in analysis results due to different personal knowledge structures, education, and experience. The analysis results are subjective, insufficient scientific, and comprehensive [8]. Therefore, considerable differences between researchers make it challenging to form a unified and authoritative research conclusion [9].

The analysis by big data-based text mining technology can improve the analysis efficiency and reduce the workload of assessment experts and researchers [10]. The big data text mining technology, advanced big data, and text analysis techniques can be used to quickly, objectively, scientifically, and comprehensively analyze the relatively mature laws on corporate social responsibility. The analysis results can help build a legal system of corporate social responsibility.

## 2. Literature Review

### 2.1. Overview of Big Data Text Mining Techniques

Big data text mining technology is a crucial technology for knowledge analysis and extraction of massive text data, which performs text data mining with the help of mature big data analysis tools [11]. New knowledge can be extracted, and basic patterns and correlations hidden in the data can be identified [12]. Big data text mining technology includes big data technology and text mining technology, which is one of the applications of big data technology in text mining [13]. Text mining based on big data can analyze the potential information of text data, discover the patterns and hidden features of text, and provide scientific and objective suggestions for the construction of corporate social responsibility legal system.

#### 2.1.1. Big Data Technology

Big data technology generally refers to tools and technologies that can acquire, process, analyze, and manage massive amounts of data [14]. Doug Laney defined the 3Vs model in a research report that classified big data technology into three dimensions: storage and analysis capacity, diversity of data, and computational speediness. As time migrated and changed, this definition was not fully applicable to all application scenarios. However, major companies like IBM, Gartner, and TechAmerica still adopted the 3Vs model in the following decade. Starting in 2011, International Data Corporation defined the 4Vs model, which summarizes the characteristics of Big Data technologies into 4Vs, namely, volume (large capacity), diversity (various forms), velocity (fast generation), and value (large values but very low density) [15]. This 4Vs model definition is now widely recognized and used.

#### 2.1.2. Text Mining Techniques

Text mining technology is an essential analytical tool and method in big data analytics [16]. Text mining is based on advanced statistics, machine learning, and linguistics techniques. It uses interdisciplinary techniques to discover patterns and trends in “unstructured data” to extract “high-quality” information [17]. Its uses include text clustering, concept extraction, sentiment analysis, and summary extraction [18]. Text mining is the process of potential mining patterns from an extensive collection of text, converting unstructured text into a structured format to identify meaningful patterns and new insights. Applying advanced analytic techniques such as Naive Bayes, Support Vector Machines (SVM), and other deep learning algorithms to explore and discover hidden relationships in unstructured data [19].

Big data provides the foundation for text mining. Text mining technology is a concrete application of big data. Only on the basis of massive text data, text mining technology can play an effective role and dig out the potential meaning.

Text mining is based on machine learning and statistical data theory to analyze and mine the implied knowledge or data collection from the text [20]. Text mining can be divided by object into data mining based on the whole text collection and data mining based on individual text. Text mining can be divided into data collection, text preprocessing, data mining, result visualization, model construction, and model evaluation according to the operation process, as shown in Figure 1.

### 2.2. LDA Theme Model

#### 2.2.1. Theoretical Basis of the LDA Model

*(1) Bayes' Theorem*. Bayes' theorem is about the conditional probability (or marginal probability) of random events A and B [21]. The theorem is that the prior probability of an event is first predicted based on previous experience [22], and then new information is obtained by other means [23]. Bayes' theorem is obtained posterior probability by correcting the prior probability with the new information [24].

The Bayesian formula is as follows.

(1) $$\begin{array}{c} P\left(A\cap B\right)=P\left(A\right)*P\left(B\left|A\right.\right)=P\left(B\right)*P\left(A\left|B\right.\right),\\ P\left(A\left|B\right.\right)=\frac{P\left(B\left|A\right.\right)\times P\left(A\right)}{P\left(B\right)}. \end{array}$$

*(2) Gibbs Sampling Algorithm*. Parameter estimation is an essential part of the LDA model. It is challenging to solve the model parameters directly, and it is necessary to use the vocabulary in the text as the observable variables. Hence, the generation of topics is the process of solving the parameters of the LDA model. There are many standard parameter inference algorithms, including EM algorithm, variational inference algorithm, and Gibbs algorithm [25]. Among them, the Gibbs sampling method is one of the Markov chain Monte Carlo methods, which is simple, efficient, and easy to implement [26]. Unknown implied variables in LDA need to be learned to estimate based on words in the observed document collection. Learning algorithms are mainly classified into exact inference and approximate inference. It has generally adopted the approximate inference algorithm to learn the implied variables in LDA, and the Gibbs sampling, as one of them, is easy to understand and has high operation efficiency. This paper adopts this method for parameter estimation. The Gibbs sampling simulates the joint distribution through conditional distribution sampling, deduces the conditional distribution through the simulated joint distribution, and iterates until it converges to the target probability distribution [27]. From the joint probability distribution *P*(*X*_0_, *X*_1_, ⋯, *X*_*n*_) to obtain *m* samples *X*^(*i*)^(*i* = 1, 2, ⋯, *m*), the method randomly initializes *X*^(0)^. For each sample, a variable *X*^(*i*)^_*j*_ can be sampled by the probability of the conditional distribution of that variable in the case of the remaining variables known *P*(*X*_*j*_^(*i*)^|*X*_1_^(*i*)^, *X*_2_^(*i*)^, ⋯, *X*_*j*−1_^(*i*)^*X*_*j*+1_^(*i*)^, ⋯, *X*_*n*_^(*i*)^), which is continuously updated to eventually form a convergent Markov chain from which samples are drawn [28]. In this paper, the process of parameter estimation using Gibbs' algorithm in the subject modelling is shown in Figure 2.

The Gibbs sampling algorithm procedure is explained as follows.

1. Initialization. *z*_*i*_(*i* = 1, 2, ..*N*)^−^ Initialized to a random integer between 1 and *T* (*T* is the number of topics).
2. Iteration. The *i* performs an iterative loop from 1 to *N*, where *N* is the number of all words in the corpus, and assigns the words to the corresponding topics according to the following equation to enter the next stage of the Markov chain

(2) $$\begin{array}{c} p\left(Z_{i}=k\left|Z_{\neg i}\right.,w_{dj},\alpha ,\beta \right)=\frac{n_{k,\neg i}^{\left(w\right)}+\beta }{\sum_{k\in \left[1,K\right]}n_{k,\neg i}^{\left(•\right)}+\beta }\cdot \frac{n_{k,\neg i}^{\left(d\right)}+\alpha }{\sum_{d\in \left[1,K\right]}n_{k,\neg i}^{\left(d\right)}-1}, \end{array}$$

where *Z*_*i*_ denotes the topic assignment of the *i*th word, *i* = *k* denotes the assignment of the randomly selected word *w* in the text to the *k*th topic as the word with subscript *i*, and *Z*_¬*i*_ denotes the topic assignment of other words besides the *i*-th word. *n*_*k*,¬*i*_^(•)^ denotes the number of words assigned to topic *k*, *n*_*k*,¬*i*_^(*w*)^ denotes the number of words assigned to topic *k* that have the same topic as *w*, and *n*_*k*,¬*i*_^(*d*)^ denotes the number of words categorized to topic *k* in the *d* text.

Iterate the second step until the smooth state of the Markov chain, taking *Z* = (*Z*_1_, ⋯, *Z*_*n*_) as a sample so that *θ* and *φ* can be obtained according to the following equation

(3) $$\begin{array}{c} {\hat{\theta }}_{k}^{\left(d\right)}=\frac{n_{k}^{\left(d\right)}+\alpha }{\sum_{k\in \left[1,K\right]}n_{k}^{\left(d\right)}+K\alpha }d,\\ {\hat{\phi }}_{k}^{\left(d\right)}=\frac{n_{\text{w}}^{\left(k\right)}+\beta }{\sum_{w\in V}n_{w}^{\left(k\right)}+N\beta }, \end{array}$$

where *n*_*w*_^(*k*)^ represents the number of times the vocabulary *w* appears in topic *k*. *n*_*k*_^(d)^ is not only the number of words containing document *d* in topic *k* but also the number of occurrences of topic *d*.

#### 2.2.2. LDA Fundamentals

LDA plays a very important role in topic model and is commonly used for text classification. It is used to speculate the topic distribution of documents, and the topic distribution of each document in the document set can be given in the form of probability distribution, so that the topic distribution can be extracted by analyzing some documents, and then topic clustering or text classification can be carried out according to the topic distribution. LDA (Latent Dirichlet Allocation) is a classical model in the generative Bayesian probabilistic model, mainly describing the process of generating text collections. Its basic idea is to view each text as a random combination of potential topics and each topic as a random combination of vocabulary [29]. The model has a three-layer Bayesian structure, including document, topic, and vocabulary layers, and is capable of mining text topics.  Figure 3 shows the structure of the model.

Document layer: document-topic distribution.

Topic layer: *ϕ* = {*Z*_1_, *Z*_2_, ⋯, *Z*_*k*_}, the set of topics for the document set, including the probabilities of individual topics and topic keywords.

Vocabulary layer: *V* = {*w*_1_, *w*_2_, ⋯, *w*_*n*_}, including all vocabulary in the document set.

The LDA model treats text as a word frequency vector and textual information as mathematical. This treatment can ignore the correspondence between words relative to documents and documents relative to document sets, converting text into probabilities, reducing the complexity of the problem, and making it easier to model [30].

The following equation shows the probability of occurrence of the words in the document after the document is generated.

(4) $$\begin{array}{c} p\left(\text{words}\left|\text{document}\right.\right)=\underset{\text{theme}}{\sum }p\left(\text{words}\left|\text{theme}\right.\right)\times p\left(\text{theme}\left|\text{document}\right.\right). \end{array}$$

Figure 4 shows the mathematical interpretation of the LDA model.

The specific mathematization of the LDA model is described as follows:

(5) $$\begin{array}{c} p\left(w,z,\theta ,\phi \left|\alpha ,\beta \right.\right)=\overset{N}{\underset{n=1}{\prod }}p\left(w_{m,n}\left|\phi \right.\right)p\left(\theta \left|\alpha \right.\right)p\left(\phi \left|\beta \right.\right). \end{array}$$

In the above formula, *K* represents the number of topics, *N*_*m*_ represents the total number of words in the *M* document, *m* represents the number of documents in the corpus, *d*_*m*_ represents the m document, *w*_*m*,*n*_ represents the *n*-th word in the *m*-th document, *z*_*m*,*n*_ represents the topic of the *n*-th word in the *m*-th document, *α* is the hyperparameter of the topic prior distribution of each document, *β* is the hyperparameter of the word prior distribution of each topic, *θm* is the topic multinomial distribution of the *m*-th document, *φk* is the word multinomial distribution of the *k*-th topic, and Dir (*α*) is the probability distribution of Dirichlet.

There are the following assumptions about the LDA model, (1) texts are independent of each other, and texts in a corpus can be exchanged. (2) The words are independent, and the words in a text can be exchanged. The document-topic distribution *θ* and the topic-word distribution *φ* in the model are random variables, which are generated using hyperparameters *α* and *β*, respectively, and the number of parameters of the LDA model is not positively correlated with the number of document sets, where the random variable *φ* obeys the Dirichlet prior distribution with *β* as the parameter.

(6) $$\begin{array}{c} \text{Dir}\left(\phi_{k}\left|\beta \right.\right)=\frac{\Gamma \left(\sum_{v=1}^{V}\beta_{v}\right)}{\prod_{v=1}^{V}\Gamma \left(\beta_{v}\right)}\overset{V}{\underset{v=1}{\prod }}\phi_{kv}^{\beta_{v}-1}, \end{array}$$

where *θ*_*kv*_ denotes the probability of vocabulary *v* in topic *k* and ∑_*v*=1_^*V*^*ϕ*_*kv*_ = 1; Γ(•) denotes the gamma (Gamma) function: Γ(*x*) = ∫_0_^∞^*t*^*x*−1^*e*^−*t*^*dt*. The other variable *θ* obeys a Dirichlet prior distribution with *α* as a parameter, i.e.,

(7) $$\begin{array}{c} \text{Dir}\left(\theta_{m}\left|\alpha \right.\right)=\frac{\Gamma \left(\sum_{k=1}^{K}\alpha_{k}\right)}{\prod_{k=1}^{K}\Gamma \left(\alpha_{k}\right)}\overset{K}{\underset{k=1}{\prod }}\theta_{mk}^{\alpha_{k}-1}, \end{array}$$

where *θ*_*mk*_ denotes the probability of topic *k* in the text *d*_*m*_ and ∑_*k*=1_^*K*^*θ*_*mk*_ = 1, for estimating parameters *θ* and *φ*; the Gibbs sampling method introduced in the previous section is chosen in this paper.

Text topics belong to the more abstract concept. Before the specific empirical application of the LDA model, the expected number of topics should be given first. Based on this and then modelling, the number of topics determined is closely related to the model analysis results. Suppose the number determined in advance is greater than the number of topics latent in the text. In that case, the model results will have redundancy, there will be invalid interfering topics if the number of topics set too small will make the topics crowded together and the exact meaning of the topics cannot be obtained, and further division is needed. In practical applications, the document set is more extensive, and the number of possible topics is also more significant. The size of the document set varies at different time stages, and the implied number of topics may be more consistent with the change in the number of document sets. Therefore, setting an optimal number of topics is crucial to the model's effectiveness before modelling the document corpus.

Many scientifically feasible methods are available today to estimate the most appropriate number of topics, such as calculating the degree of confusion and the degree of similarity between topics. In this paper, we calculate the degree of confusion to obtain the optimal number of topics. In statistical language models, the confusion degree is a standard evaluation index representing the inverse of the mean value of the similarity of all utterances in a document set, so the confusion degree is inversely proportional to the similarity degree. The specific formula is.

(8) $$\begin{array}{c} \text{Perplecity}=\exp\left\{-\frac{\sum_{m=1}^{M}\log p\left(w_{m}\right)}{\sum_{m=1}^{M}N_{m}}\right\}, \end{array}$$

where *M* refers to the set of documents, *N*_*m*_ refers to the length of the *m*th document, and *p*(*w*_*m*_) refers to the posterior probability of the *m*th document

(9) $$\begin{array}{c} p\left(w_{m}\right)=\underset{d}{\sum }\overset{N}{\underset{n=1}{\prod }}p\left(w_{j}\left|z_{j}=j\right.\right)•p\left(z_{j}=j\left|w_{m}\right.\right)p\left(d\right). \end{array}$$

The confusion is non-linearly related to the number of topics. In general, the confusion size decreases with the number of topics until the optimal number of topics is reached. The confusion value is minimized and increases with the number of topics.

### 2.3. Text Clustering

#### 2.3.1. Text Representation Model

Current text mining technology can only deal with structured data, so it is necessary to transform unstructured text into structured description [31]. Text representation means that the original text is represented by the set of feature information of the text. Textual features refer to metadata about text, which can be divided into descriptive features and semantic features. Descriptive features are easy to obtain, while semantic features are difficult to obtain. Feature representation refers to a document represented by a certain feature item (such as entry or trace). In text mining, only these feature items need to be processed, so as to realize the processing of unstructured text, which is a processing step of unstructured to structured transformation [32]. Text representation is the first step of text clustering, and there are many changes in this step, which have different effects on the final clustering effect. The common text representation models for information retrieval and text analysis include Boolean model, vector space model, and probability model.

#### 2.3.2. Selection of Feature Terms

The number of all words in the text set obtained after the separation is quite large. If they are all used as feature terms, a lot of time and resources will be wasted when performing the similarity calculation. Therefore, these words must be filtered, and the purpose of doing so is mainly two: first, in order to improve the efficiency of the program and increase the running speed: second, all words have different meanings for text classification and some general. In order to improve the classification accuracy, for each class, those words that are not very expressive should be removed and the set of feature terms for that class should be filtered. It has been demonstrated that text clustering in the feature space after feature compression degrades the clustering performance but will also help improve the clustering accuracy [33]. To extract feature information, the approach usually taken is to construct an evaluation function that evaluates against each feature and then selects a predetermined number of the best features as a subset of the resulting features according to the ranking of the feature lexicon.

#### 2.3.3. Calculation of the Weights of Feature Terms

In the vector space model, the role and importance of each feature item in the text are different, i.e., the words have different weights. The weight of a feature term integrates the contribution of that feature term to identify the text content and the ability to distinguish between texts [34]. Assuming that the size of the feature word set is *n* (i.e., there are *n* feature words), each document *D* is mapped into a vector space of dimension *n*, i.e., *V*(*D*_*j*_) = (<*T*_1_, *W*_1*i*_>, ⋯ , <*T*_*i*_, *W*_*ij*_>, ⋯ , <*T*_*n*_, *W*_*nj*_>), where *T*_*i*_(*i* ∈ [1, *n*]) denotes all the words in the feature word, and *W*_*ij*_ denotes the weight under the word in the text *D*_*j*_.

The classical definition of weights is

(10) $$\begin{array}{c} W_{ij}={{\text{TF}}_{i}}^{*}{\text{IDF}}_{j}. \end{array}$$

TF refers to term frequency, which indicates the number of occurrences of the word in document *D*, called word frequency: IDF refers to inverse document frequency, defined as

(11) $$\begin{array}{c} {\text{IDF}}_{j}=\log\left(\frac{N}{n_{j}}\right). \end{array}$$

In this formula, *N* denotes the number of all documents in the document collection, and *n*_*j*_ denotes the total number of documents in the entire document collection where the word *T*_*i*_ is present, called the document frequency of the feature.

In addition, the document length is also a factor that must be considered. Otherwise, the longer the document, the more likely it will be retrieved. The feature term weights are normalized to obtain

(12) $$\begin{array}{c} W_{ij}=\frac{{TF}_{i}\times \log\left(N/n_{j}+0.01\right)}{\sqrt{\sum_{i=1}^{m}{\left[{TF}_{i}\times \log\left(N/n_{j}+0.01\right)\right]}^{2}}}. \end{array}$$

The weight *W*_*ij*_ scales the ability of words to distinguish text content attributes. The wider the occurrence of a word in all documents, i.e., the smaller the *N*/*n*_*j*_, the smaller the *w*_*ij*_ is, indicating that its ability to distinguish document attributes is lower.

The more frequently a word appears in a particular document, the larger is *T*_*ij*_ and the larger is *W*_*ij*_, indicating that it has a stronger ability to distinguish the content attributes of the document. This formula is based on Shannon's theory of informatics. If a term appears more frequently in all texts, it contains less information entropy. If the item appears in a relatively concentrated way and only has a high frequency in a small number of texts, it will have a high information entropy.

In this way, using TF × IDF for calculation, it can get the weights of all feature words, thus completing the feature representation of the document set.

Years of experiments have shown that TF × IDF is an effective tool for text processing. This formula has been successfully applied in text classification and has promising implications for other text processing collocations, such as information distribution, filtering, and retrieval.

#### 2.3.4. Hierarchical Clustering Methods

The hierarchical clustering method generates a mesh sequence of divisions with a cluster containing all objects at the top and one cluster containing individual objects at the bottom [35]. This method decomposes a given text set at multiple levels until a specific condition is satisfied as north. Specifically, it can be divided into “bottom-up” and “top-down” methods. The “bottom-up” method is called Agglomerative Hierarchical Clustering Method (AGNES). Initially, each text is formed into a separate group. In subsequent iterations, the neighboring combinations are combined into a single group until all the texts form a single group or satisfy a specific condition. The “boot down” approach, also known as the Divisive Hierarchical Clustering Method (DIANA), is that all texts are initially organized into a group and that the group is divided into several smaller groups during the subsequent iterations until each text is in a separate group or meets some condition [36, 37]. It is shown in Figure 5.

## 3. Method

### 3.1. Corporate Social Responsibility Theme Analysis Based on the LDA Model

#### 3.1.1. Corpus Selection

The corpus data in this paper comes from the Legal Database of Peking University, which contains relevant laws and regulations from the founding of China to the present, and the content is constantly updated. It has become the most mature and professional data system for obtaining relevant documents in China. The research selects the data on laws and regulations related to corporate social responsibility.

#### 3.1.2. Constructing a Textual Syllogism Dictionary

Custom dictionaries were created based on the collected corpus texts that fit the research domain and reflect the text content. At the time of the first lemmatization, a custom lexicon had not yet been formed, and the applicability of the lemmatization results was poor. The lemmatization is inaccurate for some proper nouns, changes the meaning of the original words, or divides the words specific to the research domain into multiple universal words. Inaccurate word segmentation can seriously affect the subsequent topic mining and the analysis of the topic evolution process. Therefore, after many repeated experiments, a custom dictionary was added to the original dictionary to make word segmentation more accurate. The custom dictionary is loaded before the word-sorting operation is performed on the text during the experiment.

#### 3.1.3. Eliminating Deactivated Words

In addition to the dictionary, the construction of the deactivation lexicon also dramatically impacts the word separation effect. After using a custom dictionary, the word separation effect may still be unsatisfactory, mainly because some verbs and proper nouns with high frequency need to be removed by tools. In this study, when removing deactivated words, it first compiles a list of famous deactivated words in Chinese text: the list includes Chinese and English numbers, various punctuation marks, and a large number of words with no real meaning a lot in the text.

#### 3.1.4. Feature Selection and Vectorization

The number of words obtained by word separation and elimination of deactivated words is significant for extensive text collections. It is also necessary to filter out some high-frequency but irrelevant words for topic analysis. The TF-IDF value of the filtered data is then calculated to vectorize the data, and the use of the TF-IDF method can highlight the essential feature words and suppress the minor feature words.

Text data preprocessing is a process that needs to be repeated, continuously expanding the custom split lexicon, adjusting the deactivated lexicon, and performing feature selection based on the results until the processing results can meet the requirements of the model input. After data preprocessing, an accurate experimental corpus can be obtained.

#### 3.1.5. LDA Topic Modelling

For the LDA model, the concept of perplexity is introduced, which is an indicator to evaluate the LDA model and is used to measure the probability distribution and the quality of the model. Perplexity is the weighted average branching factor of a language, which can be interpreted as saying that if words were picked randomly at each time step from a probability distribution calculated by a language model. So on average, how many words do you have to pick to get the right one. The smaller the perplexity is, the better the quality is of the model. This paper uses the LDA Model package to model the topic model. By setting the parameter *K* and the number of iterations, it continuously adjusts the parameters to compare the weight of keywords under different topics and the size of perplexity, and finally determine the parameter *K* = 3, that is, the optimal number of topics is 5.

### 3.2. Text-Based Clustering for Corporate Social Responsibility Theme Analysis

#### 3.2.1. Determination of Initial Parameters

In *K*-average algorithm, the user is required to specify parameter *k*, and the selection of the initial *K* cluster representative objects is random, while different *K* values and different initial cluster representatives will have a great impact on the clustering quality and time efficiency, which brings many disadvantages: first, the user does not know the distribution of the clustered object set, and specifying an appropriate *K* value will add a lot of burden to the user; second, even if a suitable *k*-value is specified, the selection of the initial objects is random, which will lead to too many cycles and poor quality clustering results. Therefore, it is necessary to find the optimal number of clusters *k* by some method before using the *k*-averaging algorithm and give *k* initial objects corresponding to each cluster to obtain good time efficiency and clustering results.

This paper uses the Silhouette Coefficient-based method to determine the optimal number of clusters *k* and the density-based method to find the initial clustering centroids and combine the traditional *k*-average algorithm to achieve text clustering.

This paper uses the Silhouette Coefficient (SC) method to determine the parameter *k*, which combines cohesion and separation. Cohesion is a measure of how closely related the objects in a cluster are, and a larger cohesion indicates that the objects in a cluster are more similar. Separation measures how one cluster differs, and a smaller separation indicates that a cluster is better separated from other clusters. Generally, the maximum average contour coefficient of *K* in a small range with different values is calculated, and then the value of *K* is determined. The steps include (1) calculating and determining the range of the optimal solution 2 ≤ *k*≤$\sqrt{n}$ according to the empirical rules; (2) each value within this range is clustered by *K*-average algorithm; (3) calculate the contour coefficient of each point under different cluster number *k* and take the average value; (4) search for the maximum average contour coefficient value at different *K* and record the corresponding *K* value; (5) end of algorithm.

This paper uses a standard text classification corpus to test the initial clustering center selection effect. It contains 100 documents in 10 categories, and the clustering result should be *k* = 10. Then, *n* = 100, $\sqrt{n}$ =10, and the average contour coefficient in the 2 ≤ *k* ≤ 10 is calculated, and the test results are shown in Figure 6. With the increase of the number of clusters, Silhouette Coefficient increases gradually. When the number of clusters reaches 6, Silhouette Coefficient decreases, and then continues to increase. When KF10, Silhouette Coefficient reaches the maximum value of 0.148, which is the same as the actual number of clusters, so the value of *k* is obtained correctly.

#### 3.2.2. Selection of Initial Clustering Centers

The initial clustering centers determine the initial division of the *k*-average algorithm and greatly influence the final division. Different initial centers are chosen, and the algorithm finds different solutions. Choosing appropriate initial clustering centers can speed up the algorithm's convergence and improve the solutions' quality.

In this paper, the density method is used to determine the initial clustering centers of clusters. However, a problem arises in the actual operation process: since *r*_1_ and *r*_2_ are empirical values, for a given sample set, it is generally impossible to predict the size of *r*_1_ and *r*_2_. For *r*_2_, it can be set to a certain multiple of *r*_1_, but for *r*_1_, it is not easy to find an optimal value. *r*_1_ is too large or too small to lose the meaning of object point density and thus cannot find a reasonable initial centroid. The number of objects in the sample set, the size of each object data value, the size of each object dimension, the number of clusters *k*, the distribution of objects, and other factors will all play an important role in determining the appropriate *r*_1_ value.

This paper used the density method to determine the initial cluster center. Setting an initial value of *R*1. If the maximum density of all points is greater than 90% × *n*/*k*, subtract a step from *r*1 and recalculate the maximum density. If the maximum density of the point is less than 75% × *n*/*k*, then *r*1 is added with a step to recalculate the maximum density. In this way, the *r*1 value with the maximum density between 90% × *n*/*k* and 75% × *n*/*k* was found, so as to further determine the best clustering center point.

#### 3.2.3. *K*-Mean Based Textual Quadratic Clustering Algorithm

The above method determines the optimal number of clusters and the initial clustering centers so that the text can be clustered using the traditional *k*-average algorithm. Clustering of texts is possible using this method. However, discovering the natural number of clusters using the calculation of Silhouette Coefficient is not always effective. This drawback was found in the tests because the data may contain nested clusters for which the contour coefficient curves are not so clear.

Therefore, to address this situation, the strategy adopted in this paper is: if the number of documents contained in a cluster after clustering is more than twice that of the cluster containing the least number of documents, try to cluster the cluster again; if the cohesiveness (the sum of similarity between the objects in the cluster and the centroid) after clustering is better than the original one, split the cluster into several sub-clusters: if it is worse than the original one, keep the original cluster unchanged. In practice, it is impossible to know how many sub-clusters the clusters should be split into. In this regard, the approach taken in this paper is: for other clusters that contain similar numbers of texts, the average number of documents contained in these clusters is denoted as *q*, and the number of documents contained in the cluster to be split is denoted as *P*. The integer bit of *p*/*q* is the number of sub-clusters.

## 4. Results

### 4.1. Determining the Content of the Legal System

LDA (Latent Dirichlet Allocation) topic model can ignore the interference of textual semantic level to the text content and discover the hidden topic information in large document sets and corpus. In this paper, the LDA topic model was used for topic modelling to discover the implicit topic patterns in the text.

It can be seen from Figure 7 that at the initial stage of the growth of the number of topics, perplexity showed an obvious downward trend, and when the number of questions was 8, the perplexity was the lowest. The similarity between topics was the largest, and the generalization ability of the model was the strongest. After that, with the increase in the number of topics, perplexity shows a gradual upward trend. Hence, the optimal number of topics was determined to be 8. After determining the optimal number of topics, based on experience, the hyperparameters *α* =50/T (under the number of texts) and *β* =0.01133 are set. The Gibbs algorithm was used for the parameter estimation of *θ* and *φ*. Then, the topic modelling was performed by Python's genism library to obtain the “text-topic” distribution of the text and the probability distribution of each topic in each document. The larger the probability value of a topic in a document, the stronger the topic was in the document.

This paper used accuracy (Precision), recall (Recall), and F1-measure to judge the model effect and compared the LDA method with the W-BTM method. It can find that the LDA method had a higher effect, and the results are shown in Figure 8.

It got five corporate social responsibility themes: compliance with laws and regulations, social morality, business ethics, honesty and trustworthiness, and acceptance of supervision. Therefore, the legal system of corporate social responsibility should be built around the five aspects of compliance with laws and regulations, social morality, business ethics, honesty and trustworthiness, and acceptance of supervision.

### 4.2. Determining the Content of the Legal System

The dataset in this paper still used the standard text classification corpus, which created a folder for each of the nine major categories, and in each file, each corpus forms a text file by itself. The test sets were selected from the up-to-date corpus with different categories and different numbers of documents in each of the three test sets. For test validity, the documents in the three test sets selected in this paper are different.

This work evaluated models using accuracy (Precision), recall (Recall), equilibrium (break-evenpoint), and F1 measure (F-measure). The effect of clustering is measured using the average purity, which measures the extent to which clusters contain objects of a single class.

Let the size of the cluster *C*_*i*_ be *n*_*i*_, then the purity of the cluster is defined as

(13) $$\begin{array}{c} p\left(C_{i}\right)=\frac{1}{n_{i}}\max\left(n_{ij}\right), \end{array}$$

where *n*_*ij*_ denotes the size of the intersection of cluster *C*_*i*_ with class *j*. The average purity of the entire cluster is defined as

(14) $$\begin{array}{c} \text{purity}=\overset{k}{\underset{i=1}{\sum }}\frac{n_{i}}{n}p\left(C_{i}\right), \end{array}$$

where *k* is the number of clusters eventually formed by the clustering; the purity portrays the classification accuracy of the clustering algorithm. The higher the purity, the more effective the clustering algorithm is.

Figure 9 shows the results of the text clustering experiments based on Silhouette Coefficient and density, i.e., after the initial clustering, from which it is seen that the average purity fluctuates considerably with the size and content of the test set. The experiments again demonstrate that using Silhouette Coefficient does not guarantee the real discovery of the natural number of clusters. The *k* values determined in the experiments for test set 1 and test set 2 are 4 and 6, respectively. At the same time, the actual number of clusters is 6 and 8, which contains nested clusters, which leads to unsatisfactory clustering results. In contrast, the number of clusters *k* and the initial centroids of the test set 3 were chosen better to obtain a more uniform distribution.

To illustrate the effectiveness of the secondary clustering designed in this paper, the results after the secondary clustering of test sets 1 and 2, respectively, are shown in Figure 10, and the average purity has improved greatly, which indicates that the secondary clustering method used in this paper is effective. To further analyze the clustering effect, it listed the internal distribution of the test set with better first clustering results and the test set 1 with worse clustering results. It can be seen that clustering coalesces all documents of the same kind together and separates documents of different classes. After clustering again, the natural number of test sets is found correctly, and the results are much improved compared to the original.

Corporate social responsibility laws can be divided into five categories: social responsibility to shareholders, social responsibility to creditors, social responsibility to employees, social responsibility to consumers, and social responsibility to the environment.

### 4.3. Construction of the Legal System of Corporate Social Responsibility

The content of the legislation solves the problem of how companies assume social responsibility and how stakeholders protect their rights. According to the results of text mining, combined with the actual legal system construction principles, this paper proposes that the content of legislation focuses on the following five aspects.

Regarding social responsibility to shareholders, the protection of shareholders' right to information and the direct shareholder litigation system should be improved. Regarding social responsibility to creditors, the disclosure of company information and the early access system for creditors should be strengthened by the principle of openness. Regarding employee social responsibility, the system of employee directors and supervisors should be improved, and the tripartite consultation mechanism among the government, labor unions, and the company should be improved. Regarding social responsibility to consumers, a system for consumer participation in major corporate decisions and improving redress for damage to consumer interests should be established. Regarding social responsibility for the social environment, it should establish a system of environmental directors and establish and improve the system of environmental public interest litigation.

## 5. Discussion

This study used big data text mining technology to analyze legal texts and achieved rapid, efficient, scientific, and objective effects. However, the sample data collected is not enough; the training set in Chinese words, high-frequency word dictionaries, and other datasets are insufficient, and the analysis results may not be comprehensive enough.

Future research should collect more sample data to ensure the comprehensive analysis results of the social responsibility legal system. Since the relevant legal text data are mainly in Chinese, the analysis method based on big data text mining technology designed in this study only applies to Chinese and translated text mining. It lacks the mining algorithm design for original English text data. Future research should add English text data mining algorithm to make big data text mining algorithm suitable for Chinese and English text data mining. At the same time, in the research process, topic discovery and text clustering will be subject to subjective influence to a certain extent, and the research results are related to the personnel's knowledge background and cognitive ability. In future research, a set of evaluation criteria is needed to evaluate the research results to exclude human factors.

## 6. Conclusion

Corporate social responsibility is a research field that has the connotation of The Times and has great development potential. There are many disciplinary perspectives and research methods in related research. However, the research methods remain in traditional qualitative research, lacking quantitative, objective, and accurate research. After theme analysis and text clustering of legal corpus data by text mining method, the results were obtained to put forward five aspects of the legal system construction framework, which is used to guide the construction of the corporate social responsibility legal system. This study breaks through the traditional method of constructing the legal system based on expert experience and used a large amount of corpus text to mine the legal theme and content, and found the potential legal system framework, which had a certain pioneering significance.

## Figures and Tables

**Figure 1:** Text mining flowchart.

**Figure 2:** Gibbs sampling parameter estimation process.

**Figure 3:** LDA model three-layer structure diagram.

**Figure 4:** Directed probability model diagram of LDA model.

**Figure 5:** Schematic diagram of hierarchical clustering algorithm.

**Figure 6:** Average Silhouette Coefficient under different *k* values.

**Figure 7:** Number of topics-perplexity.

**Figure 8:** Comparison of the effect of LDA and W-BTM theme models.

**Figure 9:** The results of text clustering based on Silhouette Coefficient and density.

**Figure 10:** The results of secondary clustering of test sets 1 and 2.

## Data Availability

The analyzed datasets generated during the study are available from the corresponding authors on reasonable request.
